The article "Looking for Responders among Women with Chronic Pelvic Pain Treated with a Comicronized Formulation of Micronized Palmitoylethanolamide and Polydatin" was published in 2022. Journal: Biomed Res Int.

# Looking for Responders among Women with Chronic Pelvic Pain Treated with a Comicronized Formulation of Micronized Palmitoylethanolamide and Polydatin

**DOI:** 10.1155/2022/8620077

**Published:** 2022-05-07

**Authors:** Ugo Indraccolo, Alessandro Favilli, Arianna Dell'Anna, Antonio Di Francesco, Barbara Dionisi, Emilio Giugliano, Filippo Murina, Erica Stocco

**Affiliations:** ^1^Maternal-Infantile Department, Complex Operative Unit of Obstetrics and Gynecology, “Alto Tevere” Hospital of Città di Castello, ASL 1 Umbria, Via L. Angelini 10, 06012 Città di Castello, Italy; ^2^Maternal-Infantile Department, Section of Obstetrics and Gynecology, Azienda Ospedaliera Universitaria Integrata di Verona, Hospital of Woman and Child, Piazzale Stefani 1, 37126 Verona, Italy; ^3^Obstetrics and Gynecology Unit, “Santa Caterina Novella” Hospital of Galatina ASL Lecce, Via Roma, 73013 Galatina, Italy; ^4^Obstetrics and Gynecology Unit, “Floraspe Renzetti” Hospital of Lanciano, ASL 2 Abruzzo, Via per Fossacesia 1, 66034 Lanciano, Italy; ^5^“Santa Famiglia” Health House of Rome, Via dei Gracchi 134, 00192 Roma, Italy; ^6^Maternal-Infantile Department, Complex Operative Unit of Obstetrics and Gynecology, “Santa Maria della Misericordia” Hospital of Rovigo ULSS 5 Veneto, Viale Tre Martiri 140, 45100 Rovigo (PD), Italy; ^7^Obstetrics and Gynecology Department Lower Genital Tract Disease Unit “Vittore Buzzi” Hospital University of Milano, Via Castelvetro 32, 20154 Milano, Italy; ^8^Vulvodynia Italian Association, Via G.B. Pergolesi 4, 20124 Milano, Italy; ^9^Department of Surgical, Oncologic and Gastroenterologic Sciences, First Surgical Clinic, University of Padua, Via Giustiniani 2, 35128 Padova, Italy

## Abstract

**Background:**

Palmitoylethanolamide is reported to solve pain and neuroinflammation in different models of chronic and neurodegenerative diseases. Some concerns have been illustrated for cautiously interpreting the available literature on the topic. Specifically, there is a lack of evidence about palmitoylethanolamide and female chronic pelvic pain. Concerns will be best solved by randomized trials. The present study was aimed at finding the best responders to micronized palmitoylethanolamide in female patient with chronic pelvic pain, using the existing literature at individual patient level, to help further randomized trial planning.

**Methods:**

After a systematic research, eligible studies (the ones enrolled female patients treated for chronic pelvic pain or for dyspareunia, dysuria, dyschezia, and dysmenorrhea with or without chronic pelvic pain) were assessed at individual patient data level. Conditional probabilities were calculated to assess variables conditioning the rates of good responders (pain score points more or equal to 3 reduction), poor responders (2 pain score reduction), and nonresponders at a three-month follow-up.

**Results:**

Only cases treated with palmitoylethanolamide comicronized with polydatin for a short period can be assessed. Good responders are more than 50%. In chronic pelvic pain, there is a 19.0% conditional probability to find good responders among patients with pain score at enrolment of 6 to 8 and of 6.8% to find poor responders among patients with a pain score at enrolment of 6 to 8. Painful disease does not matter on responders' rates.

**Conclusion:**

Best responders to comicronized palmitoylethanolamide/polydatin are patients with pain score higher than 6 at enrolment, irrespective of other variables.

## 1. Introduction

Chronic pelvic pain is a common problem that affects mainly the female population, and it is caused by a dysfunction, damage, or degeneration of the sensory nervous system. This condition leads to a significant discomfort and reduction of the patient quality of life [1].

In recent years, scientific literature has expressed positive opinions about palmitoylethanolamide (PEA). While mast cells and glia cells are acknowledged having pivotal role in chronic inflammatory disorders [2–4], PEA is able to block persistent activation of these cells [5], thereby playing an important role in the resolution of pain and neuroinflammation in different models of chronic and neurodegenerative diseases [6].

The mechanism of action of PEA has been recently summarized by D'Amico et al. [7]. First, it acts as an “ALIA” molecule able to directly downregulate mast cell degranulation. Second, it activates at least two nuclear receptors, the peroxisome proliferator-activated receptor alpha (PPAR*α*) and the orphan receptor G-protein coupling (GPR55), provoking a somewhat regulation of the proinflammatory behaviour of the cell. Third, PEA plays a so-called entourage action, by enhancing the anti-inflammatory and anti-nociceptive function of other substances (among them, the ones involved in activating the cannabinoid receptors 1 and 2).

The strength points of PEA naïve along with hypothetical weakness have been exposed in several reviews, on the base of experimental data and clinical issues [8–14]. Micronized and ultramicronized palmitoylethanolamide (m-PEA and um-PEA) have been used for preclinical and clinical studies to overcome the concern of PEA bioavailability. Both m-PEA and um-PEA are constituted by a crystalline form with a particle size between 100 and 700 *μ*m [15] characterized by a high surface-volume ratio that allows a better diffusion, distribution, and higher biological efficacy compared to nonmicronized PEA [16, 17]. In 2016, however, Gabrielsson et al. [9] suggested to cautiously interpret the available literature on PEA because of a conflict of interest issue and poor-quality clinical trials. Specifically, the issue of PEA and chronic pelvic pain is still poor to date, while more data have been provided for chronic pain, as reported by Paladini et al. [18] in pooled data meta-analysis.

In a previous aggregate data meta-analysis on female patients with pelvic pain [19], the authors have proved that m-PEA comicronized with transpolydatin (Pol) allows a significant reduction of pain scores in female patients with endometriosis suffering from chronic pelvic pain.

Transpolydatin (Pol) is a natural glucoside of resveratrol, an antioxidant and anti-inflammatory molecule. Pol has been combined with m-PEA in a comicronized form (9 mg of m-PEA and 1 mg of Pol) [m(PEA/Pol)]. Besides endometriosis [19–22], m-PEA/Pol has been used in the treatment of interstitial cystitis/bladder syndrome [23] and dinitrobenzene sulfonic acid- (DNBS-) induced colitis [24].

The U. Indraccolo et al. meta-analysis [19] was unable to detect a subgroup of patients able to show a larger pain reduction, although it suggested that the higher the pain score at enrolment, the greater the pain reduction. Additionally, meta-analyzed data [19] do not report how many responders to the m(PEA/Pol) have been found and if such reduction can be observed in chronic pelvic pain patients with other painful diseases. Moreover, it is unknown if the effectiveness observed in the U. Indraccolo et al. [19] meta-analysis is due to m-PEA, Pol, or both. Understanding how many patients would be responders to m-PEA and if a subgroup of best responders exists among them is needed to plan hypothetical randomized trials on the compound efficacy.

Compounds with PEA and Pol formulations (both associated and alone) are commercialized in some countries as foods for special medical purpose (with heterogeneous regulatory issues [25]). Therefore, in some countries, they can be administered in spite of lacking of registrative trials supporting their efficacy, the route of administration, and their dosage.

The present study was aimed at finding the best responders to m-PEA in female chronic pelvic pain patients, using the existing literature at individual patient level.

## 2. Methods

A systematic review was planned and registered in the PROSPERO database (CRD42021232156).

The best responders to m-PEA are planned to be assessed in a descriptive way, by pooling individual data from databases of already published articles on the topic. No comparators are planned to be assessed in the present work.

### 2.1. Systematic Research

In December 7, 2020, a systematic review was drawn on PubMed, Web of Science, Scopus, SciELO, African Journal Online, and Asian Digital Library. The search on each database was done using the following MeSH: palmitoylethanolamide AND chronic pelvic pain; palmitoylethanolamide AND pelvic pain; palmitoylethanolamide AND endometriosis; and palmitoylethanolamide AND dysmenorrhoea. Neither time frame nor language limits were set. Already published systematic reviews and meta-analyses on PEA [18, 19, 26, 27] were also screened for collecting more references on PEA clinical series. More articles were collected by screening the Epitech Group SpA database on spontaneous studies on m-PEA.

Prospective and retrospective studies, randomized trials, and clinical descriptive series, where an arm of cases was treated with m-PEA, were all screened for eligibility at individual patient level.

Eligible studies were the ones in which female patients were treated for chronic pelvic pain or other pelvic pain with or without chronic pelvic pain (even in a subgroup of the sample). After the screening phase of the studies selection (Figure 1), the corresponding authors, of the 11 references [20, 22, 23, 28–36] eligible for inclusion, were contacted to share their full databases by mail or phone. Those databases would be judged eligible for a further analysis if they had at least one case of a female patient with at least a pelvic pain reported as dysmenorrhea, dysuria, dyschezia, dyspareunia (irrespective from deep or superficial dyspareunia or both), and chronic pelvic pain.

Pain had to be assessed with the visual analogue scale (VAS) or numeric rating scale (NRS). Pain had to have a value score point of 5 or more at enrolment in one or more of the above-mentioned pains and had to be assessed in a three-month follow-up for the same pain. Any other information useful for assessing the characteristics of responders was planned to be collected from single databases.

Responders were defined as patients reporting a reduction of pain, from enrolment to three-month follow-up, of 2 or more scores in one or more symptoms of chronic pelvic pain as dysmenorrhea, dyspareunia, dyschezia, and dysuria. Among responders, we also differentiated poor responders (only 2 VAS or NRS score point reduction from the enrolment value at the three-month follow-up) from good responders (3 or more VAS or NRS score points reduction from the enrolment value at the three-month follow-up).

### 2.2. Data Synthesis

Cases with no pain score at enrolment of 5 or more in none of the pains were excluded from the whole pooled case database. Rates of good responders, poor responders, and non responders were calculated on the whole. Then, rates of nonresponders, poor responders, and good responders were reported for chronic pelvic pain, dysmenorrhea, dyspareunia, dyschezia, and dysuria groups.

A conditional probability of occurrence of each patient characteristics (independent variables) extracted from the pooled case database among nonresponders, poor responders, and good responders at three-month follow-up was also provided.

### 2.3. Statistical Analysis

The pooled case database has been assessed by principal component two-dimensional correspondence analysis for each type of pain: dysmenorrhea, dysuria, dyschezia, dyspareunia, and chronic pelvic pain. The two dimensions were organized among the dependent variables (nonresponders, poor responders, and good responders at three-month follow-up) and all other independent variables theoretically involved in pain perception. Those independent variables were extracted at individual patient level. The correspondence analysis output provides a two-axis map with dependent and independent variables summarized as points with proper coordinates. The higher is the closeness of the independent variables to the point dependent variables, the higher their association. Therefore, by calculating distances among points, it is possible to estimate the unconditioned probabilities of associations of variables. The distances were rescaled to be between 0 and 1, as probability does. Finally, by applying Bayes' theorem, the conditional probability was calculated for each independent variable and each group of responders for all types of pain. Associations are hypothesized if conditional probabilities are found to be more than 0.05 (5%), setting the *P* value for chance of less or equal to 0.05. Therefore, the higher is the probability over the 0.05, the higher the strength of association.

As a complimentary analysis, the percentage of association among good responders and no good responders of each type of pelvic pain with chronic pelvic pain was checked. Such analysis is needed as chronic pelvic pain sensitization can increase pain perception for other pains with acute behaviour.

IBM SPSS 27 was used for principal correspondence analysis, and LibreOffice 7.0 was used to perform other calculations.

### 2.4. Quality Assessment

A modified GRADE score [37] was used to assess the quality of data, in relation with the specific methodology used for performing the present study. The aim of this scoring system is to give an overall objective judgment of the quality of the available databases for meeting the aims of the current study, as poor-quality study has been reported to be a practical concern in interpreting the literature on PEA [9]. We did not plan to exclude poor studies from the review, as the main aim of the study was not to demonstrate any superiority of m-PEA.

The modified GRADE scoring system has been:

1. Type of study: +3 for randomized series, +2 for prospective observational series, +1 for retrospective series, and 0 for small series (less than 5 cases)
2. Availability of descriptive data for calculating unconditional probabilities: +3 full items available; +2 more than a half of items available; +1 less than a half of items available; and 0 no additional information than pain score at enrolment and at three months follow-up available
3. Numerosity of the eligibility series: +1 if more or equal to 10 and -1 if less than 10
4. Presence of comparator arm: -1: no comparator arm and 0: comparator arm is reported, but the quality assessment of the study provided by the Newcastle-Ottawa [38] scale (for observational studies) or by the Jadad et al. [39] scale (for randomized studies) is less than a half of maximum score; +1: comparator arm is reported, and the quality assessment of the study provided by the Newcastle-Ottawa [38] scale (for observational studies) or by the Jadad et al. [39] scale (for randomized studies) is more than, or equal to, a half of maximum score.

The score was attributed by UI and AF. In case of no agreement, discussion among UI and AF led to the final score.

To each pooled case, it was assigned the score given to the study where such case was extracted. The pooled scores were averaged for each kind of subgroup of pain (chronic pelvic pain, dysmenorrhea, dyspareunia, dyschezia, and dysuria). The scoring system of the study can vary from -2 to 8, with mean value of 3. For single subgroup series of pooled data, a quality mean score of more than 3 indicates that the quality is higher than the mean. The mean quality has been provided for each subgroup of pain, along with 95% confidence intervals (CI).

## 3. Results

Figure 1 reports the phases of systematic review in a flow chart. Studies eligible by viewing the full database were 11, but full databases have been shared by only 7 authors of studies [20, 22, 29–32, 34]. One hundred seventeen cases were collected. According to the inclusion criteria, 24 cases were excluded because patients did not have at least one pain score at enrolment of 5 or more in at least a type of pain. Therefore, 93 pooled cases were assessed.

Table 1 reported the characteristics of each study assessed for inclusion. None of these studies provides data on patients treated with m-PEA alone. All studies reported data on the association of m-PEA/Pol. Quality score attributed to each study is reported in Table 2.

Sixty-four patients had chronic pelvic pain of 5 or more (68.8%), 28 (30.1%) had dyspareunia (unspecified if deep or superficial or both), 15 (16.1%) dyschezia, 19 (20.4%) dysuria, and 34 (36.6%) dysmenorrhea. The quality score for pooled cases is slightly higher than 3 (Table 3). Table 3 reports also the crude numbers and rates of good responders, poor responders, and nonresponders according to each type of pain at the three-month follow-up.

Among available additional information in databases, 10 items have been extracted: patient' age at enrolment, years of pains, years elapsed from pains onset to diagnosis of painful disease, type of painful disease (endometriosis, vulvodynia, and unknown or unreported painful disease), menopausal status, previous surgery, use of analgesics during treatment, hormonal therapies during treatment, transcutaneous electrical nerve stimulation (TENS), and pain value at enrolment. These items were assessed as independent variables.

Figure 2 illustrates the conditional probability of each type of independent variables for the five types of pain (dysmenorrhea, dysuria, dyschezia, dyspareunia, and chronic pelvic pain) for good responders, poor responders, and nonresponders at the three-month follow-up.

In chronic pelvic pain, there is a 19.0% conditional probability to find good responders among patients with pain score at enrolment of 6 to 8; there is a conditional probability of 6.8% to find poor responders among patients with a pain score at enrolment of 6 to 8. Poor responders have a 41.8% conditional probability to use analgesics. The conditional probability that nonresponders associate with any of the variables reported in Figure 2 is less than 5% (not significant). Additionally, the type of painful disease does not matter on responders' rates.

In the dysmenorrhea and dysuria group (Figure 3), good responders, poor responders, and nonresponders are not found to be associated to any of the variables assessed. In dyspareunia group (Figure 3), good responders have a conditional probability of 20.6% to undergo TENS, while in the dyschezia group (Figure 3), good responders have a conditional probability of 5.7% to be found among patients with pain score at enrolment of 6 to 8 and of 13.0% to be found among patients with pain score at enrolment of more than 8. Again, the type of painful disease does not matter on responders rates.

Finally, Table 4 reports the percentage of concordance among number of improvement or no-improvement in at least one acute pain and chronic pelvic pain at the three-month follow-up. The concordances observed are all over 50%.

## 4. Discussion

The present review was aimed at finding the best responder female patient to the m-PEA in chronic pelvic pain. Instead, basing on the available literature, the work is able to find the best responder female patient to short-duration treatment with PEA comicronized with Pol at the three-month follow-up, assessing more variables available at individual patients slides. Prior to initiate a randomized trial, such a kind of study would be advisable, to know the proportion of patients needed to be enrolled to obtain an appropriate sample size and their characteristics.

Ninety-three heterogeneous patients had any type of pelvic pain (pain score equal to or more greater than 5). More than 50.0% of them have a very good improvement (3 pain score points or more) of their pain in at least one pain item, and more than 70% are overall responders at the three-month follow-up. All these patients have been treated with m-(PEA/Pol) for two months or more. The improvement of pain scores is not affected by type of painful disease, proving that m-(PEA/Pol) acts on pain and not on the specific painful disease. Those results were achieved from individual patient series with intermediate quality score, extracted from 7 studies of low quality at aggregate level. Five out of 7 studies have not any comparator arm and are not blinded. In our opinion, this is the higher concern as placebo efficacy is a well-known bias for pain killer drugs assessment, sometimes hard to control in clinical trials on pains [40].

In chronic pelvic pain and dyschezia groups of patients, we found that the best responders at the three-month follow-up to the m-(PEA/Pol) therapy are the ones with pain score at enrolment of more than 6. Additionally, good responders to dyspareunia, dysmenorrhea, dysuria, and dyschezia are likely to be good responders also to chronic pelvic pain (Table 4), thereby confirming that pain control by m-(PEA/Pol) would be exerted on pain sensitization [41]. On the other hand, no other factors than higher pain score at enrolment has been linked with pain reduction at the three-month follow-up, excluding the TENS treatment for dyspareunia and the use of analgesics for chronic pelvic pain in poor responders patients.

Therefore, in planning a hypothetical randomized trial aiming to prove the efficacy of the m-(PEA/Pol) combination, chronic pelvic pain of more than 6 pain score point cases should be enrolled. Arranging both a placebo arm and a no-treatment arm [40] would be advisable for ruling out the efficacy of the placebo from the hypothetical efficacy of the m-(PEA/Pol). In all these hypothetical arms, the consumption of analgesics has to be assessed.

The present review does not exclude that poor responders to the m-(PEA/Pol) at the three-month follow-up would be able to become good responders after more than three-month therapy. Poor responders seem being 10-25% (Table 3). The experimental design of the reviewed studies available in literature are mainly focused on a three month follow-up. Therefore, further data on more than three months therapy are needed. Additionally, dyspareunia has been assessed without considering deep or superficial dyspareunia complained by patients with endometriosis or vulvodynia. TENS has been only administered to patients with vulvodynia in the Murina et al. study [32], explaining why good responders in the dyspareunia group associate with TENS treatment. While the specific localization of dyspareunia was not reported in the pooled case database, it is likely that good responders to the combination complained of superficial dyspareunia, as superficial dyspareunia is complained in vulvodynia cases.

A limitation of the study comes from missing information from unavailable databases. It would be very interesting to assess unavailable databases [23, 28, 33, 35, 36] at individual patient level because missing studies assess the effectiveness of m-(PEA/Pol) in painful bladder syndrome/interstitial cystitis [23, 33], primary dysmenorrhea [38], and more painful cases of endometriosis [28, 35]. All these studies demonstrate significant improvement of pain. The Tartaglia et al. study [36] and the Cobellis et al. [28] study are also randomized trials. The results would suggest a good degree of efficacy for m-(PEA/Pol) along with very good effectiveness.

A further limitation of the present study is that the number of pooled patients with pain is low for pelvic pains of acute behaviour (dyspareunia, dysmenorrhea, dyschezia, and dysuria). Therefore, number of cooccurrence of chronic pelvic pain and other type of pain is very low, as reported in Table 4. While the probabilistic approach to the analysis does not need many data, a randomized trial would take into consideration that cooccurrence of chronic pelvic pain, and other types of pelvic pain, is an uncommon event.

As no data has been registered in chronic pelvic pain for m-PEA without Pol, it is still unclear how effective is the combination of m-(PEA/Pol) versus single micronized agent administration (specifically, the m-PEA). m-PEA has been reported to be effective for other kinds of chronic pain [42]. The item should be a matter of further investigation.

Quite stringent criteria for quality assessment could lead to underrating some study basing on a questionable subjective view. The step is needed for being as soon honest as possible for the interpretation of the available literature at individual patient level, thereby addressing the issue of poor-quality studies exposed by Gabrielsson et al. [9]. Moreover, the individual patient approach is able to overcome the confusion between effectiveness and efficacy of PEA.

In conclusion, short-duration treatments with m-(PEA/Pol) would allow an improvement of pain score in chronic pelvic pain patients of 3/4 of cases. Half of treated patients would improve by at least 3 points of pain score, while 1/4 would improve of 2 points of pain score. The improvement is not conditioned by any painful disease. Best responders in chronic pelvic pain are patients with pain score at enrolment between 6 and 8. Other acute pelvic pains (dyspareunia, dyschezia, dysuria, and dysmenorrhea) would benefit from treating chronic pelvic pain. These evidences came from low-quality study and from pooled case databases of intermediate quality. They strongly suggest that efficacy and effectiveness of the m-(PEA/Pol) short-time treatments for chronic pelvic pain in female patients have to be proved against placebo and no-treatment in randomized trial.

## Figures and Tables

**Figure 1:** Flow chart of the phases of systematic review.

**Figure 2:** Conditional probabilities to be good responders, poor responders, and nonresponders for each variables assessed in chronic pelvic pain group.

**Figure 3:** Conditional probabilities to be good responders, poor responders, and nonresponders for each variables assessed in dysmenorrhea, dyschezia, dyspareunia, and dysuria groups.

**Table 1:** Description of studies of which databases has been assessed at individual patient level. Included cases are reported in the last column at the right side.

	Treatment	Disease	Pain assessment	Enrolment	Eligible cases	Included cases
Dell'Anna and De Marzi [29]	Um-PEA 200 mg m-(PEA/Pol) 400 mg/40 mg 3 times daily for four months	Endometriosis	NRS	Prospective	Single arm: 16	14
Di Francesco and Pizzagallo [22]	m-(PEA/Pol) 400 mg/40 mg two times daily for six months	Endometriosis	NRS	Randomized	An arm: 10	9
Dionisi and Senatori [30]	m-(PEA/Pol) 400 mg/40 mg two times daily for two months, plus topical adelmidrol	Vulvodynia/vestibulodynia	NRS	Prospective	Single arm: 34	17
Giugliano et al. [31]	m-(PEA/Pol) 400 mg/40 mg two times daily for three months	Endometriosis	VAS	Prospective	Two arms (but no comparator arm): 19 and 28	15 and 18
Indraccolo and Barbieri [20]	m-(PEA/Pol) 400 mg/40 mg two times daily for three months	Endometriosis	VAS	Small series	4 cases	4
Murina et al. [32]	m-(PEA/Pol) 400 mg/40 mg two times daily for two months	Vestibulodynia	VAS	Randomized	An arm: 10	9
Stocco and Schievano [34]	m-(PEA/Pol) 400 mg/40 mg two times daily for two months	Miscellaneous symptoms	VAS/NRS	Prospective	Single arm: 13 (male and female)	7

m-PEA: micronized palmitoylethanolamide; um-PEA: ultramicronized palmitoylethanolamide; Pol: polydatin.

**Table 2:** Quality score given for each study.

	Type of study	Availability of descriptive data	Numerosity of the series	Presence and appropriateness of comparator arm	Total score of the study
Dell'Anna and De Marzi [29]	2	2	1	-1	4
Di Francesco and Pizzagallo [22]	3	2	-1	0	4
Dionisi and Senatori [30]	2	2	1	-1	4
Giugliano et al. [31]	2	2	1	-1	4
Indraccolo and Barbieri [20]	0	3	-1	-1	1
Murina et al. [32]	3	2	-1	1	5
Stocco and Schievano [34]	2	2	-1	-1	2

No observational study with comparator arm has been found (so the Newcastle-Ottawa scale was not applied). The Giugliano et al. [31] study is a two-arm study; both arms are treated with the m-(PEA/Pol).

**Table 3:** Quality score attributed at individual patient level (first column, left side). Additionally, the unconditional probabilities of good responders, poor responders, and nonresponders are reported as crude numbers and rates, according with type of pain.

	Nonresponders	Poor responders	Good responders
Chronic pelvic pain (*N* = 64) -Quality score: 3.6 (3.4-3.8)	14 (21.9%)	17 (26.6%)	33 (51.6%)
Dysmenorrhea (*N* = 34) -Quality score: 3.9 (3.7-4.1)	6 (17.6%)	3 (8.8%)	25 (73.5%)
Dyspareunia (*N* = 28) -Quality score: 4.0 (3.6-4.4)	3 (10.7%)	2 (7.1%)	23 (82.1%)
Dyschezia (*N* = 15) -Quality score: 3.5 (3.0-4.0)	3 (20.0%)	2 (13.3%)	10 (66.7%)
Dysuria (*N* = 19) -Quality score: 3.8 (3.5-4.2)	1 (5.3%)	0	18 (94.7%)

**Table 4:** Rates of concordances among chronic pelvic pain and other type of pain of acute behaviour.

	Good responders in both	No good responders in both	Percentage of association
Dysmenorrhea and chronic pelvic pain (*N* = 19)	9	8	17/19 89.5%
Dyspareunia and chronic pelvic pain (*N* = 16)	9	3	12/16 75.0%
Dyschezia and chronic pelvic pain (*N* = 14)	5	5	10/14 71.4%
Dysuria and chronic pelvic pain (*N* = 8)	3	3	6/8 75.0%

## Data Availability

The articles cited for the organizing database [16, 18, 24–27, 29] report the corresponding authors' names and contacts. Authors can be contacted for information on data.
